The article "Reducing motion artifacts in 4D MR images using principal component analysis (PCA) combined with linear polynomial fitting model" was retracted in 2015. Reasons: fabricated or falsified data; concerns about the data.

# Reducing motion artifacts in 4D MR images using principal component analysis (PCA) combined with linear polynomial fitting model

**DOI:** 10.1120/jacmp.v16i2.5165

**Published:** 2015-03-08

**Authors:** Juan Yang, Hongjun Wang, Yong Yin, Dengwang Li

**Affiliations:** ^1^ School of Information Science and Engineering, Shandong University Jinan Shandong China; ^2^ Department of Radiation Oncology Shandong Cancer Hospital and Institute Jinan Shandong China; ^3^ School of Physics and Electronic Science, Shandong Normal University Jinan Shandong China

**Keywords:** motion artifacts, linear polynomial fitting, principal component analysis, 4D MRI, motion trajectory

## Abstract

We have previously developed a retrospective 4D‐MRI technique using body area as the respiratory surrogate, but generally, the reconstructed 4D MR images suffer from severe or mild artifacts mainly caused by irregular motion during image acquisition. Those image artifacts may potentially affect the accuracy of tumor target delineation or the shape representation of surrounding nontarget tissues and organs. So the purpose of this study is to propose an approach employing principal component analysis (PCA), combined with a linear polynomial fitting model, to remodel the displacement vector fields (DVFs) obtained from deformable image registration (DIR), with the main goal of reducing the motion artifacts in 4D MR images. Seven patients with hepatocellular carcinoma (2/7) or liver metastases (5/7) in the liver, as well as a patient with non‐small cell lung cancer (NSCLC), were enrolled in an IRB‐approved prospective study. Both CT and MR simulations were performed for each patient for treatment planning. Multiple‐slice, multiple‐phase, cine‐MRI images were acquired in the axial plane for 4D‐MRI reconstruction. Single‐slice 2D cine‐MR images were acquired across the center of the tumor in axial, coronal, and sagittal planes. For a 4D MR image dataset, the DVFs in three orthogonal direction (inferior–superior (SI), anterior–posterior (AP), and medial–lateral (ML)) relative to a specific reference phase were calculated using an in‐house DIR algorithm. The DVFs were preprocessed in three temporal and spatial dimensions using a polynomial fitting model, with the goal of correcting the potential registration errors introduced by three‐dimensional DIR. Then PCA was used to decompose each fitted DVF into a linear combination of three principal motion bases whose spanned subspaces combined with their projections had been validated to be sufficient to represent the regular respiratory motion. By wrapping the reference MR image using the remodeled DVFs, ‘synthetic’ MR images with reduced motion artifacts were generated at selected phase. Tumor motion trajectories derived from cine‐MRI, 4D CT, original 4D MRI, and ‘synthetic’ 4D MRI were analyzed in the SI, AP, and ML directions, respectively. Their correlation coefficient (CC) and difference (D) in motion amplitude were calculated for comparison. Of all the patients, the means and standard deviations (SDs) of CC comparing ‘synthetic’ 4D MRI and cine‐MRI were 0.98±0.01,0.98±0,01, and 0.99±0.01 in SI, AP, and ML directions, respectively. The mean±SD Ds were 0.59±0.09 mm,0.29±0.10 mm, and 0.15±0.05 mm in SI, AP and ML directions, respectively. The means and SDs of CC comparing ‘synthetic’ 4D MRI and 4D CT were 0.96±0.01,0.95±0.01, and 0.95±0.01 in SI, AP, and ML directions, respectively. The mean±SD Ds were 0.76±0.20 mm,0.33±0.14 mm, and 0.19±0.07 mm in SI, AP, and ML directions, respectively. The means and SDs of CC comparing ‘synthetic’ 4D MRI and original 4D MRI were 0.98±0.01,0.98±0.01, and 0.97±0.01 in SI, AP, and ML directions, respectively. The mean±SD Ds were 0.58±0.10 mm,0.30±0.09 mm, and 0.17±0.04 mm in SI, AP, and ML directions, respectively. In this study we have proposed an approach employing PCA combined with a linear polynomial fitting model to capture the regular respiratory motion from a 4D MR image dataset. And its potential usefulness in reducing motion artifacts and improving image quality has been demonstrated by the preliminary results in oncological patients.

PACS numbers: 87.57.cp, 87.57.nj, 87.61.‐c

## I. INTRODUCTION

Four‐dimensional computed tomography (4D CT) has been widely used to monitor patient‐specific respiratory motion for determining individual safety margin in radiation therapy.^1^, ^2^, ^3^, ^4^, ^5^ However, 4D CT does not provide sufficient breathing motion information of soft tissue due to low soft‐tissue contrast, and imposes substantial ionizing radiation dose to the patient due to increased image acquisition time.^6^, ^7^, ^8^ As an alternative, MRI‐based 4D imaging techniques, which are able to capture sufficient motion information of soft‐tissue and involve no ionizing hazard, are highly desirable in clinic.^(9)^

Currently, many 4D‐MRI techniques have been proposed mainly containing two approaches:^10^, ^11^, ^12^, ^13^, ^14^, ^15^, ^16^, ^17^ 1) using a 3D MR sequence to acquire real‐time volumetric images (i.e., real‐time 4D MRI); and 2) using a fast 2D MR sequence to continuously acquire images from all respiratory phases and retrospectively sort these images according to the respiratory phases (i.e., retrospective 4D MRI). However, to acquire high‐resolution 4D MR images using the first approach is difficult due to the limitations of current available hardware and software. Compared to the real‐time 4D MRI, the retrospective approach can acquire MR images with high image quality using respiratory surrogate to monitor the patients' respiratory motion during image acquisition. Hu et al.^(16)^ proposed a prospective 4D‐MRI technique using triggers at preselected respiratory amplitude to acquire T2‐weighted MR images. This amplitude‐based technique has the advantage of improving the tumor‐to‐tissue contrast‐to‐noise ratio (CNR) by acquiring T2‐weighted 4D‐MRI image datasets, and it is more robust to irregular breathing compared to phase‐based 4D‐MRI. Tryggestad et al.^(17)^ presented a novel retrospective 4D‐MRI technique to acquire a longer duration MRI to derive the average or most probable state of mobile anatomy and meanwhile capture and convey the observed motion variability. The respiratory phase bins for sorting the dynamic MRI frames were derived from postprocessing the respiratory signals. Two‐pass approaches in retrospective sorting were used to acquire ‘De‐blurred’ 4D MRI. Currently, we also developed a retrospective 4D‐MRI technique using body area (BA) as an internal respiratory surrogate.^(9)^ Preliminary results in liver cancer patients have demonstrated the feasibility and fidelity of this technique.^(10)^ However, unavoidable artifacts in the reconstructed 4D MR images were observed. Those artifacts were presumably caused by irregular respiratory motion which were commonly observed in 4D CT,^(18)^ and dark phase dispersion bands and ghost artifacts using FIESTA/TrueFISP sequences for image acquisition. Besides, inaccurate calculation of respiratory phases also contributed to the artifacts.^(19)^

Many studies related to reducing motion artifacts have been proposed.^20^, ^21^, ^22^ Liao et al.^(20)^ presented an approach of reducing motion artifacts in dynamic cardiac MRI by increased sampling density in certain regions of the k‐space spanning most of the energy of the inconsistencies. Several variable‐density spiral trajectories were designed and tested, and their efficiencies for reducing motion artifacts were evaluated in computer simulations and healthy volunteers. The authors concluded that variable‐density spiral trajectories could effectively reduce motion artifacts with a small loss in signal‐to‐noise ratio (SNR) as compared in uniform density counterpart. Nehmeh et al.^(21)^ proposed a method referred to as respiratory‐correlated dynamic PET (RCDPET) to reduce respiratory motion artifacts in PET images of lung cancer. The authors compared this method with respiratory‐gated PET (RGPET) and concluded that the RCDPET was comparable method to RGPET in reducing artifacts caused by respiration and improving the image quality of PET in thorax. However, the RCDPET had an advantage over the RGPET of reconstructing PET image at any phase or amplitude in breathing cycle. Zhang et al.^(22)^ presented a patient‐specific motion modeling to reduce motion artifacts in 4D CT images caused by irregular motion during 4D CT acquisition. Principal component analysis (PCA) was used to reconstruct the motion vectors obtained from deformable image registration (DIR). The authors demonstrated that the regular motion of a subject could be accurately represented by three principal motion bases and their projections. The synthesized CT images with reduced motion artifacts were reconstructed by deforming the reference CT image using the reconstructed motion vectors. The motion modeling was evaluated in three lung cancer patients and the results demonstrated the high efficiency of the proposed approach in reducing severe image artifacts.

In this work, inspired by the investigation of Zhang et al., we proposed a method employing PCA to reduce the motion artifacts in 4D MRI. But the different point between the two studies was that a supplementary process of fitting the displacement vector fields (DVFs) was added in our study, with the main goal of correcting the registration errors caused by 3D registration algorithm. The DVFs between the reference image and the phase images of 4D MRI were calculated using an in‐house DIR algorithm. A linear polynomial fitting method was used to fit the DVFs in three temporal and spatial dimensions to correct the potential registration errors, and then PCA was employed to decompose the fitted DVF in each direction into linear combination of three principal motion bases, whose spanned subspaces had been validated to be able to represent the regular respiratory motion of a patient. By wrapping the reference MR images with the reconstructed DVFs, the ‘synthetic’ MR images at selected phase were synthesized. The preliminary results of liver and lung cancer patients demonstrated that the proposed method could be used for reducing irregular motion artifacts in 4D MRI without much loss of respiratory motion information.

## II. MATERIALS AND METHODS

### A. Patient cohort and imaging study

Eight patients (3 male, 5 female, mean age of 68.0 yrs) who had liver cancer(s) (7/8) or lung cancer (1/8) were enrolled in this IRB‐approved prospective study. The patients' clinical characteristics are summarized in Table 1. All patients underwent MR and CT scans on the same day for treatment planning.

For each patient, a 4D CT scan was performed under uncoached free breathing condition on a 16‐slice CT scanner (Philips Brilliance Bores CT; Philips Healthcare, Andover, MA) equipped with Real‐time Position Management (RPM) system (Varian Medical Systems, Inc., Palo Alto, CA) and Advantage 4D software (GE Healthcare, Milwaukee, WI). The respiratory signal was recorded with the RPM gating system by tracking the trajectory of infrared markers placed on the patient's abdomen. Each CT image from the scanner was labeled by the time tag according to the respiratory signal. The reconstructed 4D CT images were sorted into 10 respiratory phases based on tags by the Advantage 4D software, with 0% corresponding to end‐inhalation and 50% corresponding to end‐exhalation. The imaging parameters were as following: voltage/current: 120 kV/290 mA, slice thickness: 2.5 mm, gantry rotation: 0.5 s per cycle, reconstruction matrix: 512×512, field of view (FOV): 450–500 mm.

**Table 1:** Summary of patients' characteristics and measurements

*Patient*	*Age*	*Gender*	*Cancer Site*	*Scanner Type*	*‘Synthetic’ 4D MRI vs. cine‐MRI ‘Synthetic’ 4D MRI vs. 4D CT ‘Synthetic’ 4D MRI vs. original 4D MRI*					
					*CC*		*D (mm)*		
					*SI*	*AP*	*ML*	*SI*	*AP*	*ML*
1	52	M	HCC	1.5 T	0.98 0.96 0.98	0.99 0.96 0.98	0.99 0.95 0.98	0.50 0.55 0.46	0.25 0.30 0.30	0.12 0.10 0.13
2	68	F	Liver Mets	1.5 T	0.98 0.95 0.98	0.97 0.95 0.97	0.99 0.96 0.96	0.60 0.70 0.62	0.28 0.32 0.32	0.05 0.08 0.10
3	70	F	HCC	3.0 T	0.97 0.97 0.99	0.98 0.96 0.98	0.99 0.94 0.98	0.62 1.00 0.65	0.50 0.60 0.50	0.20 0.30 0.22
4	72	M	HCC	3.0 T	0.99 0.96 0.98	0.97 0.94 0.97	0.98 0.93 0.97	0.40 0.50 0.45	0.13 0.10 0.18	0.15 0.20 0.18
5	78	F	Liver Mets	1.5 T	0.99 0.95 0.99	0.98 0.95 0.99	0.99 0.94 0.96	0.70 1.05 0.72	0.30 0.30 0.25	0.20 0.22 0.22
6	65	F	Liver Mets	1.5 T	0.97 0.96 0.98	0.98 0.94 0.98	0.99 0.96 0.97	0.58 0.78 0.60	0.25 0.40 0.32	0.20 0.20 0.18
7	68	F	Liver Mets	3.0 T	0.98 0.97 0.96	0.97 0.95 0.98	0.98 0.97 0.98	0.60 0.81 0.65	0.32 0.30 0.28	0.18 0.22 0.15
8	70	F	NSCLC	3.0 T	0.99 0.98 0.99	0.99 0.96 0.97	0.99 0.95 0.98	0.55 0.68 0.50	0.30 0.32 0.29	0.12 0.16 0.15
Mean	68	/	/	/	0.98 0.96 0.98	0.98 0.95 0.98	0.99 0.95 0.97	0.59 0.76 0.58	0.29 0.33 0.30	0.15 0.19 0.17
SD	7.5	/	/	/	0.008 0.01 0.01	0.008 0.008 0.007	0.005 0.01 0.009	0.09 0.20 0.10	0.10 0.14 0.09	0.05 0.07 0.04

MR simulations included a 4D‐MRI scan and single‐slice cine MR scans. All MR scans were performed on a 1.5 Tesla (Signa, GE Healthcare, Milwaukee, WI) or a 3.0 Tesla MR system (MAGNETOM Trio, Siemens Healthcare, Erlangen, Germany) using a fast steady state acquisition imaging technique (labeled as FIESTA by GE and TrueFISP by Siemens). No immobilization device was used during image acquisition. Multiple‐phase MR images were acquired in the axial plane, including multiple slices to cover a volume of interest. Scan time per axial slice was set to approximately two to three times the patient's breathing period. Single‐slice 2D cine MR images were acquired across the center of the tumor in three orthogonal (axial, coronal, and sagittal) planes for 30 s using the same sequence as the 4D‐MRI scan. MRI parameters were optimized to achieve fast image acquisition (>3 frames/s) while maintaining adequate spatial resolution: repetition time (TR)/echo time (TE): 3.005 ms /1.128 ms; FOV: 300∼480×360∼480 mm; flip angle: 50°; slice thickness: 5 mm; bandwidth: 976.562 Hz/pixel; acquisition matrix: 192×128. MRI images were interpolated to 256×256 before further analysis.

### B. 4D MRI reconstruction

The retrospective 4D MRI technique using BA as the respiratory surrogate was utilized to reconstruct the coronal and sagittal MR images. The feasibility of this technique has been validated in our previous publication^9^, ^10^ and we will briefly describe this technique here.

To determine the breathing signal, each MR image was first processed to determine the body contour. BA used as the respiratory surrogate in the 4D‐MRI technique, was defined as the number of pixels within body contour. Individual breathing curve at each slice location was then generated by plotting the BA as a function of image acquisition time. The complete breathing signal was obtained by combining individual breathing curves continuously according to the image acquisition time, followed by removing the low frequency component of the signal, which was caused by anatomical changes. The low frequency component was generated using low‐pass filter, and the low frequency was set to 5–10 Hz.

To reconstruct the 4D MRI, an automatic search algorithm was used to detect respiratory peaks from the complete breathing signal, followed by a manual correction to remove erroneous peak detections. Peaks were assigned to Phase 50% and linear interpolation was used to calculate the rest of the phases. In cases where a phase was missing, the nearest phase and corresponding MR image were used to reconstruct the 4D MRI. Two‐dimensional cine MR images were retrospectively rebinned into 10 phases according to respiratory phases. In addition, the first two images in the image series at each slice location were excluded for reconstruction, which allowed for the MR signals reaching a steady state (i.e., consistent signal). All image processing and data analysis were performed using an in‐house programming implemented in MATLAB (MathWorks Inc., Natick, MA).

### C. Deformable registration across 4D MR images

The DVFs from MR images at a reference phase to all the other phase images were obtained using an in‐house DIR algorithm based on B‐spline implemented in a commercial software (Velocity AI 2.4; Velocity Software Inc., Mountain View, CA), which has been validated as an accurate and robust method.^(23)^ In this study, without loss of generality, MR images at the first phase (T=0%) were used as the reference image for all patients. MR‐corrected deformable registration algorithm accompanied with the determination of region of interest (ROI) was used to tackle with the alignment between the secondary images (the phase images) and the primary image (the reference phase). Then the DVFs were automatically calculated during the registration procedure and were exported for analysis. Figure 1 showed the workflow of generating ‘synthetic’ 4D MRI using our method based on linear polynomial fitting model and PCA in this study.

**Figure 1:** Workflow of generating the ‘synthetic’ 4D MRI using our method. Firstly, displacement vector fields (DVFs) are obtained from the deformable image registration (DIR) between a reference MR image and other phase images. Secondly, DVFs are fitted in three temporal and spatial dimensions using a linear polynomial fitting model. Thirdly, the principal component analysis (PCA) is utilized to decompose each of the DVF into linear combinations of principal motion bases whose spanning subspaces are validated sufficient to capture the major variations of respiratory motion. Finally, the ‘synthetic’ 4D MRI is generated by deforming the reference MR image using the reconstructed DVFs.

### D. Remodeled DVFs reconstruction

#### D.1 DVFs fitting using linear polynomial fitting model

As aforementioned, an in‐house DIR algorithm was used to solve the alignment problem in this study. The DVFs were calculated by deforming all the phase images to the reference image (T=0%) respectively, and a drawback of the 3D DIR was that it did not consider the continuity of the displacements of each pixel at corresponding phases throughout the respiratory cycle. To correct the registration errors introduced by 3D DIR, a linear polynomial fitting model was utilized to fit the displacement trajectory of each pixel. Then the same polynomial was used to fit the displacements of adjacent pixels at each phase in three spatial dimensions to correct the potential discontinuous motion introduced by temporal fitting. Thus the total DVF fitting (F) was composed by temporal fitting ($F_{t}$) and spatial fitting ($F_{s}$) with corresponding weights, which was denoted by

(1) $$F=\lambda F_{t}+(1-\lambda )F_{s}$$

where parameter λ indicted the weighting of temporal fitting ($F_{t}$), and (1−λ) was the weighting of spatial fitting ($F_{s}$). The weighting factor λ used for balancing the spatial fitting and the temporal fitting was chosen through trials in our study. Different values of λ as 0.6, 0.7, 0.8, and 0.9 have been substituted to Eq. (1), respectively, since we wanted to focus on the temporal fitting. The results demonstrated that good temporal fitting as well as good spatial fitting could be obtained using the value of 0.8 for λ.

For a 4D MR image data, the DVFs can be represented by triplet of matrices, denoted by D={Dx,Dy,Dz}, where Dx, Dy, and Dz are the 3D DVF matrices in the medial–lateral (ML), anterior–posterior (AP), and superior–inferior (SI) directions, respectively. Without any loss of generality, we used the DVF matrix in the SI direction (Dz) to detail the fitting work in this study, which was also applicable for the other two directions.

The displacement field (Dz) was columnwise vectorized, mathematically, and was denoted as $Dz=\{\vec{d}(1),\vec{d}(2),\ldots ,\vec{d}(N)\}(P\times N)$, consisting of N (N=10) displacement fields, where $\vec{d}(2),\vec{d}(3)$. and $\vec{d}(10)$ represented the displacement vectors between the reference image (T=0%) and the phase images (T=10%,20%…… and 90%), respectively, and $\vec{d}(1)$, denoted as the displacement field between the reference phase (T=0%) and the phase images (T=0%), was structured as a zero matrix with the same size as the other column vectors. As shown in Fig. 1, to avoid the problem of solving large system of equations, the high‐dimensional matrix Dz was down‐sampled into a low‐dimensional matrix $Dz^{\prime }$ with a size of L×N (L<P). Then we used a quartic polynomial which had been found to provide sufficient flexibility and spatial accuracy to fit the low‐dimensional $Dz^{\prime }$ by row‐wise and by column‐wise, which represented the DVF fitting in temporal dimension and spatial dimension, respectively. The same polynomial was used to fit the DVF matrices in ML and AP directions, respectively. The final fitted DVFs in three orthogonal directions were obtained for the next step of analysis.

#### D.2 Motion artifacts reduction for4D MRI using PCA

To capture respiratory motion signals from the noisy DVFs and reduce motion artifacts in the 4D MR images, PCA was used to find the major motion bases in the respiratory motion. Firstly, the covariance matrix of the fitted DVF was calculated, given as

(2) $$Cov=\frac{1}{N-1}{\sum_{i=1}^{N}\left(\vec{d^{\prime }}(i)-\vec{\bar{d}})(\vec{d^{\prime }}(i)-\vec{\bar{d}}\right)}^{T}$$

where ${\vec{d}}^{\prime }(i)$ indicated the fitted column vector between the phase image at the ith phase and the reference image, and the vector $\vec{\bar{d}}$ represented the mean of those column vectors, given as

(3) $$\vec{\bar{d}}=\sum_{i=1}^{N}\vec{d^{\prime }}(i)$$

The purpose of this step was to find an optimal transformation that mapped the high‐dimension space to a low‐dimension subspace, with the minimum of the mean‐square error. By solving the eigenvalues and eigenvectors of the variance matrix *Cov*, the transformation could be readily obtained. We could use Eq. (4) to solve the eigenvalues and eigenvectors:

(4) $$Cov\lambda_{j}=\lambda_{j}{\vec{\varphi }}_{j}$$

where $\lambda_{j}$ and ${\vec{\varphi }}_{j}$ were the jth eigenvalue and the corresponding eigenvector of matrix *Cov.* The transformation matrix *Φ* ___was generated by concatenating all the nonzero eigenvalues of matrix *Cov,* sorted in descendent order according to their corresponding eigenvalues, as $\Psi =\{{\vec{\varphi }}_{1},{\vec{\varphi }}_{2},{\vec{\varphi }}_{3},\ldots ,{\vec{\varphi }}_{p}\}(p\leq 10)$, satisfying $\lambda_{1}\leq \lambda_{2}\geq \ldots \geq \lambda_{p}\;{\vec{\varphi }}_{j}$ was the direction of basis vector, and $\lambda_{j}$ was the corresponding variance along this direction. Then the *n* principal motion bases were decided by satisfying

(5) $$\lambda_{1}+\lambda_{2}+\ldots +\lambda_{n}\gg \sum_{j=n+1}^{N}\lambda_{j}$$

The equation indicated that the principal motion bases ${\vec{\varphi }}_{1},{\vec{\varphi }}_{2},{\vec{\varphi }}_{3},\ldots ,{\vec{\varphi }}_{n}$ might be sufficient to capture the major variations of deformable motion in the liver or lung, thus the transformation matrix can be described by these principal motion basis vectors. In our study, it was observed that the sum of first three eigenvalues dominated and account for ∼85% of total variations from eight oncologic patients. Then ${\vec{d}}^{\prime }(i)$ could be represented by three projection coefficients onto low‐dimension subspaces spanned by the principal motion bases ${\vec{\varphi }}_{1},{\vec{\varphi }}_{2}$ and ${\vec{\varphi }}_{3}$. The projection coefficients were calculated as

(6) $$\begin{array}{l} \theta_{1}(i)={\vec{\varphi }}_{1}^{T}({\vec{d}}^{\prime }(i)-\vec{\bar{d}})\\ \theta_{2}(i)={\vec{\varphi }}_{2}^{T}({\vec{d}}^{\prime }(i)-\vec{\bar{d}})\\ \theta_{3}(i)={\vec{\varphi }}_{3}^{T}({\vec{d}}^{\prime }(i)-\vec{\bar{d}}) \end{array}$$

In this study, three principal motion bases and corresponding projection coefficients were used to reconstruct the original fitted DVF in each direction, thus significant dimension reduction was realized without much loss of major motion information. Figure 2 (top left) shows the eigenvalues of the covariance matrix in SI direction from the 4D MR image set of Patient #1. The trajectories of projection coefficients corresponding to the first five bases were displayed in Fig. 2 (top right and bottom row). The trajectory motion of projection coefficients onto the first three bases (Fig. 2 top right) were obvious, but the other two trajectories showed tiny motion (Fig. 2 bottom row). The results implied that the principal motion bases captured the regular respiratory motion, while the rest of the bases might be account for minor variations, such as noises derived from image artifacts or errors caused by DIR. So the reconstruction of original fitted DVFs was calculated from the Eq. (6), using

(7) $$\hat{\vec{d}}(i)=\vec{\bar{d}}+\theta_{1}(i){\vec{\varphi }}_{1}^{T}+\theta_{2}(i){\vec{\varphi }}_{2}^{T}+\theta_{3}(i){\vec{\varphi }}_{3}^{T}$$

**Figure 2:** Results of principal component analysis (PCA) on DVFs in superior–inferior (SI) direction for Patient #1: (top left) eigenvalues; (top middle and top right) the trajectory of projection coefficients onto 1st and 2nd eigenvectors; (bottom) the trajectory of projection coefficients onto 3rd (left), 4th (middle), and 5th (right) eigenvectors.

The above analysis was also applicable for DVFs in AP and ML directions. So the reconstructed DVFs in each direction could be approximately represented by the linear combination of three principal motion bases with the ability of capturing the major respiratory motion. The reconstructed DVFs were retrospectively interpolated into original size for the reconstruction of ‘synthetic’ 4D MRI.

### E. Reconstruction of ‘synthetic’ 4D MRI

As mentioned, the principal motion bases containing less noise introduced by the errors of DIR could be used to represent the regular respiratory motion. Therefore, the reconstructed DVFs contained less noise caused by the registration errors in DIR. The ‘synthetic’ MR images with reduced artifacts at each phase were generated by deforming the reference MR image (T=0%) using the reconstructed DVFs calculated in Eq. (7). As shown in Eq. (7), the reconstructed DVFs at phase *i* was denoted by $\vec{d}(i)$, and the MR image $I_{i}$ at phase *i* could be obtained by wrapping the MR image $I_{ref}$, at the reference phase, described by

(8) $$I_{i}({\vec{X}}_{i})=I_{ref}(\vec{X}+\vec{d}(\vec{X},i)$$

where $\vec{X}$ represents a voxel's location in the reference MR image $I_{ref}$, and ${\vec{X}}_{i}$ stands for the voxel's location in the MR image $I_{i}$ at phase *i*.

### F. Comparison of 4D tumor motion trajectories

Cine‐MRI, 4D CT, and original 4D MRI were used to validate the motion accuracy of ‘synthetic’ 4D MRI. For the single‐slice, cine‐MRI and three 4D images, tumor motion trajectories in three orthogonal directions (SI, AP, and ML) were extracted from the images using an automatic tracking algorithm based on cross‐correlation.^24^, ^25^, ^26^ Notably, there were differences between the cine MR used here and the other one used for 4D MRI. The single‐slice, cine‐MR imaged only one slice across the center of the tumor in three orthogonal directions (SI, AP, and ML). Whereas, the multiple‐slice, cine‐MR used for 4D MRI was acquired in the transverse plane.

Coronal and sagittal 4D‐MRI images were reconstructed. In order to compare tumor motion trajectories determined from the ‘synthetic’ 4D MRI, each of the tumor motion trajectories of the single‐slice, cine‐MRI was processed to generate average tumor motion trajectories containing only one breathing cycle. Tumor trajectories in the SI and AP directions were extracted from sagittal images (for both 4D and cine) and were extracted from coronal images (for both 4D and cine) in the ML direction. Although we could also acquire the SI tumor motion information from coronal images, that information was not used due to the concern of errors caused by through‐plane (i.e., AP) tumor motion. For sagittal MR images, the through‐plane (i.e., ML) tumor motion is less concerning since tumor motion in the ML direction is typically very small. The tracking process was repeated five times for each 4D CT and 4D MRI in order to remove human variations in selecting the base template that was used for tracking. Using repeated measurements to determine the average tumor motion trajectories can eliminate this human variation.

Tumor motion trajectories determined from cine‐MRI, 4D CT, original 4D MRI, and ‘synthetic’ 4D MRI were then compared. Since the cine‐MRI was acquired near real‐time relative to the tumor motion, it was used as the reference for evaluating the tumor motion measurement of ‘synthetic’ 4D MRI. Specifically, the correlation coefficient (CC) and the difference in motion amplitude (D) between the motion trajectories were calculated for each patient. The difference in motion amplitude, D, was calculated as the mean difference in amplitude of the 10 respiratory phases between cine‐MRI, 4D CT, original 4D MRI, and ‘synthetic’ 4D MRI.

## III. RESULTS

### A. Phantom study

To validate the feasibility of our proposed method, we acquired 4D‐MRI images of a phantom.^(9)^ The cylindrical imaging object made from gel was programmed to undergo sinusoidal motion with a 5 s period and a peak‐to‐peak amplitude of 20 mm. A fiducial marker was placed into the central of the imaging object. Multiple‐phase, multiple‐slice 2D MR images was acquired using a clinical 1.5 T scanner (Signa, GE Healthcare, Milwaukee, WI) using a FIESTA sequence. MR imaging parameters were: repetition time (TR)/echo time (TE): 3.2 ms/1.0 ms; field of view (FOV): 300×300 mm; flip angle: 50°; slice thickness: 5 mm; matrix: 192×128; frame rate: 3 frames/s. And the 4D‐MR images were reconstructed using the BA as the respiratory surrogate. Single‐slice 2D cine‐MRI was also imaged in the sagittal plane across the center of the imaging object using the same MR sequence (FIESTA) as used in 4D MRI and the same imaging parameters. Since cine‐MRI acquires near real‐time images, it was used to obtain the true motion of the phantom in the SI direction. The motion trajectory of the phantom determined from the cine‐MRI served as a ground truth, and was compared with that determined from the 4D MRI.

Software of Velocity AI was used to perform registration between the reference image and other phase images, with the MR images at Phase T=0% selected as the reference. The DVFs were remodeled using the polynomial fitting model and the PCA analysis. The ‘synthetic’ 4D MRI was reconstructed using the remodeled DVFs.

Figure 3 shows original (Fig. 3(a)) and ‘synthetic’ (Fig. 3(b)) 4D MRI. Figure 4 shows the comparison of the motion trajectories of the imaging object determined from the sagittal 4D MRI and the sagittal cine‐MRI. It was obvious that the image quality of the ‘synthetic’ 4D MRI were improved compared with the original 4D MRI with comparable respiratory motion as cine‐MRI. The mean (± standard deviation (SD)) D between the two was 0.28±0.5 mm.

**Figure 3:** Original (a) and ‘synthetic’ (b) 4D MR images. It was obvious that the image quality of the ‘synthetic’ 4D MRI were improved compared with the original 4D MRI.

**Figure 4:** Comparison of the motion trajectories of the imaging object determined from the sagittal 4D MRI and the sagittal cine‐MRI. The mean absolute difference (±SD) in motion amplitude between the two was 0.28±0.5 mm.

### B. Patient study

5, 8 show the representative results of Patient #1. Figure 5 shows the comparison of 3D displacement trajectories of a pixel over one breathing cycle before (a) and after (b) temporal fitting using a linear polynomial fitting model. The results demonstrated that the motion trajectory became smooth after the fitting scheme.

To evaluate the accuracy of the polynomial fitting method used in this study, we compared tumor motion trajectories before/after the fitting (recorded by DVFs) with the tumor motion trajectory derived from the cine‐MRI (real time) (shown as Fig. 6). From the figure, we can see that the motion after fitting was closer to the real‐time motion, and the D between DVFs after fitting and cine‐MRI was smaller than 0.22 mm, compared to 0.35 mm between DVFs before fitting and cine‐MRI.

Figure 7 shows the comparison of DVFs in the sagittal plane before (Fig. 7(a)) and after (Fig. 7(b)) spatial fitting using the same linear polynomial fitting model as the temporal fitting. The lines indicated the displacement profiles in a specific row before and after spatial fitting.

Figure 8 shows an example of original 4D MRI (shown as Fig. 8(a)) and ‘synthetic’ 4D MRI (shown as Fig. 8(b)) in sagittal plane. The arrows indicated the image artifacts. The diaphragm structures in the original 4D MRI at some phases were severely distorted; however, it was observed that both the shape and the structural information were restored near the diaphragm and the image quality was improved as well due to the wrapping procedure using the remodeled DVFs.

Figure 9 shows the comparison of original 4D MRI (Fig. 9(a)) and ‘synthetic’ 4D MRI (Fig. 9(b)) from the lung cancer patient. It was obvious that the distorted regions indicated by the red arrows in the original 4D MRI were greatly restored in the ‘synthetic’ 4D MRI using our proposed method.

**Figure 5:** The displacement trajectories of a pixel in three dimensions throughout the respiratory cycle before (a) and after (b) temporal fitting using a linear polynomial fitting model in Patient #1.

**Figure 6:** Comparison of tumor motion trajectories derived from DVFs before/after fitting and the tumor motion from cine‐MRI (real‐time) in orthogonal directions (SI, AP, and ML).

**Figure 7:** Comparison of DVFs in the sagittal plane in a specific slice before (a) and after (b) spatial fitting using a linear polynomial fitting model. The lines indicted the displacement profiles.

Figure 10 shows the comparison of tumor motion trajectories between cine‐MRI, 4D CT, original 4D MRI, and ‘synthetic’ 4D MRI. Good matching was observed between cine‐MRI and ‘synthetic’ 4D MRI: the CC ranged from 0.98 to 0.99 and the D ranged from 0.05 mm to 0.60 mm, with the largest value in the SI direction. Good agreement was also found between 4D CT and ‘synthetic’ 4D MRI: the CC ranged from 0.93 to 0.96 and the D ranged from 0.08 mm to 1.05 mm. Good matching was also observed between original 4D MRI and ‘synthetic’ 4D MRI: the CC ranged from 0.96 to 0.99 and the D ranged from 0.10 to 0.72.

**Figure 8:** Representative 4D MRI before (a) and after (b) the presented method. It is visible that artifacts distorted the original 4D MRI, but the distorters are mitigated in the ‘synthetic’ 4D MRI.

**Figure 9:** Comparison of original 4D MRI (a) and ‘synthetic’ 4D MRI (b) from the lung cancer patient. It was obvious that the distorted regions indicated by the red arrows in the original 4D MRI were greatly restored in the ‘synthetic’ 4D MRI using our proposed method.

Table 1 summarizes the measurement results of all the patients. Of all the patients, the means and SDs of CC comparing ‘synthetic’ 4D MRI and cine‐MRI were 0.98±0.01,0.98±0.01, and 0.99±0.01 in SI, AP, and ML directions, respectively. The mean±SD Ds were 0.59±0.09 mm,0.29±0.10 mm, and 0.15±0.05 mm in SI, AP, and ML directions, respectively. The means and SDs of CC comparing ‘synthetic’ 4D MRI and 4D CT were 0.96±0.01,0.95±0.01, and 0.95±0.01 in SI, AP, and ML directions, respectively. The mean±SD Ds were 0.76±0.20 mm,0.33±0.14 mm, and 0.19±0.07 mm in SI, AP and ML directions, respectively. The means and SDs of CC comparing ‘synthetic’ 4D MRI and original 4D MRI were 0.98±0.01,0.98±0.01, and 0.97±0.01 in SI, AP, and ML directions, respectively. The mean±SD Ds were 0.58±0.10 mm,0.30±0.09 mm, and 0.17±0.04 mm in SI, AP, and ML directions, respectively.

**Figure 10:** Comparison of tumor motion trajectories from cine‐MRI, 4D CT, and original and ‘synthetic’ 4D MRI in orthogonal directions (SI, AP, and ML). Error bars are standard deviations of multiple measurements in 4D CT, original 4D MRI, and ‘synthetic’ 4D MRI and are standard deviations of multiple breathing cycles in cine‐MRI. Each of the 30 s long tumor motion trajectories of the single‐slice cine MRI was processed to generate average tumor motion trajectories containing only one breathing cycle for motion comparison.

## IV. DISCUSSION

In this work we represented a mathematical method which combined a linear polynomial fitting model and PCA to reduce motion artifacts in original 4D MRI. Tumor motion trajectories derived from cine‐MRI, 4D CT, original 4D MRI, and ‘synthetic’ 4D MRI were compared to validate the motion accuracy of ‘synthetic’ 4D MRI, with the results indicating that the presented method could be used for reducing motion artifacts without much loss of respiratory motion information. The original 4D MRI was reconstructed with our proposed 4D‐MRI technique, using body area as the respiratory surrogate. However, the source MR images were acquired using a fast imaging sequence employing steady‐state acquisition (FIESTA). So a potential disadvantage of this technique is the suboptimal tumor‐to‐tissue, contrast‐to‐noise ratio (CNR) due to the T2*/T1 weighting mechanism of the sequence (compared to T2 weighting), which may affect the accuracy of DIR. In addition, the wrapping approach requires at least one 3D MR image at a specific phase with high image quality to hold the post of reference image, and the quality of ‘synthetic’ MR images will be compromised if artifacts exist in the reference image, as shown in Fig. 11.

In the study by Zhangand colleagues,^(22)^ the authors used an in‐house developed dual‐force “demons” algorithm to obtain DVFs from CT images at a reference phase to CT images at all the other phases of a 4D CT dataset. It was obvious that the prerequisite condition for modeling respiratory motion was accurate DVFs acquisition. Benchmark sets were used to evaluate the accuracy of the DIR algorithm in Zhang's study. However, the potential errors introduced by out of considering the continuity of displacements of each pixel at 10 phases in the 3D DIR algorithm for 4D CT images registration were not taken into consideration. Compared with Zhang's method, the represented approach in our study incorporated the procedure of fitting DVFs in three temporal and spatial dimensions using polynomial fitting model, which could potentially correct the registration errors in 3D DIR algorithm. In addition, in the Zhang study, they did not positively validate the efficiency of their continuous respiratory motion, since only the reconstructed CT images at the original phases (T=0%,10%, ….., and 90%) were compared with corresponding CT images without comparing the CT images at reconstructed phases, such as T=5%,28%,98%, etc. This might be mainly due to lack of ground truth. However, a drawback of our method was that the presented approach used to reduce the motion artifacts was performed through patient‐by‐patient in three orthogonal directions (SI, AP, and ML) instead of modeling the respiratory motion to retrospectively reconstruct continuous respiratory motion. Therefore, limited phase stamps were reconstructed throughout a respiratory cycle in our study. It is of great interest to develop a patient‐specific motion modeling as Zhang and colleagues did, to enhance the flexibility of our study in future investigation. In addition, PCA^(27)^ was used in both studies to capture the respiratory motion signals from the displacement field. However, to our best knowledge, it is difficult to remove image noise without loss of useful information. PCA is used here to map the original high‐dimensional space onto a low‐dimensional subspace and to capture the principal motion bases that can be used to characterize the regular respiratory component. Although those “minor variations” may contain some regular motion, they are a fraction of the total. Three principal motion bases with corresponding projections were validated sufficient to represent the regular respiratory motion in our study demonstrated by the final results. In addition, it was observed that a subspace spanned by one principal motion base with its projection were validated to be sufficient to represent the DVF in each direction in the Zhang study, whereas three principal motion bases with corresponding projections were used to reconstruct the DVFs in each direction in our study, which has been validated sufficient to represent the regular respiratory motion. This might be due to the differences in respiratory motion patterns, image acquisition modes or DIR algorithms used in the two studies.

**Figure 11:** Example of 4D MRI before (top row) and after (bottom row) our proposed method. Distortions (indicted by red arrows) still exist in the ‘synthetic’ 4D MRI due to poor image quality of the reference image.

This pilot study included a limited number of patients and assessed only by patients with intrahepatic cancer. A larger pool of patients is needed in future studies in order to answer the following questions: 1) How does the irregular respiratory motion affect the performance of our method? 2) Is this method effective to cancers in other locations treated by radiation therapy, such as esophageal cancers? 3) Are there any other methods to better demonstrate the accuracy of respiratory motion in the ‘synthetic’ 4D MRI?

In the DVFs fitting process, on the one hand, the polynomial was decided, not only to warrant a good agreement with the original data in three orthogonal directions (SI, AP, and ML), but also to keep the trajectories smooth and reasonable. It may be more rational to select patient‐specific and direction‐specific polynomial by considering respiratory motion patterns, cancer locations, and different motion amplitudes in three orthogonal directions. However, for the sake of simplicity, we used the same polynomial for DVFs fitting in ML, AP, and SI directions for all patients, which might introduce potentially insufficient fitting or over‐fitting for the DVFs. On the other hand, in order to accelerate the processing speed and avoid out of memory, the DVFs in three orthogonal directions were down‐sampled into a small size and then retrospectively interpolated into original size after the fitting and PCA procedures. All data analysis and image processing were performed in MATLAB 2012b (MathWorks), installed in a computer with Intel(R) Core(TM) i7‐3770 CPU @ 3.40GHz, RAM of 8.00G, and 64‐bit operating system. Considering the limitation of available hardware and balancing between avoid solving a large system of equation and information/resolution loss, the typical value of L in this study was chosen as 128×128×30 after several trials compared with the typical value of P as 256*256*30. The DVFs remodeling process typically consumed 5 min for each patient. So this may introduce potential errors to the reconstructed DVFs by regarding as the neighboring voxels having displacements with linear changes. But in practice, there are nonlinear changes in the displacements of adjacent voxels due to irregular respiratory motion pattern.

Many interesting results on the use of PCA for modeling respiratory motion have been reported. Zhang et al.^(28)^ found that the regular respiratory motion of a specific patient could be accurately represented by using of the first two principal bases. And their motion model was used to correct the motion artifacts in 4D CT and daily cone beam CT (CBCT). In their study, the DVFs in each direction were concatenated and then stacked into a big matrix. Li et al.^(29)^ proposed a method for understanding of PCA on the modeling of the spatial‐temporal relationship of the motion for lung. Although PCA is a useful and attractive method to map the high‐dimension space to a low‐dimension subspace, it does not separate the high‐order or nonlinear components which may affect the PCA‐based calculation by the mean‐square approximation.^(22)^ Independent component analysis (ICA), which is used to find the independent components (also called factors, latent variables or sources) by maximizing the statistical independence of the estimated components, is the most extensively studied technique among many other techniques for high‐dimensional data. The ICA can achieve the high‐order independence by decomposing the high‐dimensional space into statically independent components with different weights. In the field of multivariate statistics, kernel principal component analysis (kernel PCA)^(30)^ is an extension of PCA, using techniques of kernel theory which has drawn great attention and has shown some potential. The kernel PCA has been demonstrated to be useful for novelty detection^(31)^ and image denoising.^(32)^ Using a kernel, the originally linear operations of PCA are done in a reproducing kernel Hilbert space with a nonlinear mapping. He et al.^(33)^ proposed a method for estimating the patient‐specific CTs at random phases using a static 3D CT and the real‐time respiratory signals of that patient, who did not generally take 4D CTs. The kernel PCA (K‐PCA) was used for establishing a motion estimation model, which was constructed to estimate the lung field motion from the fiducial motion using the ridge regression method based on the least squares support vector machine. So it will be worthwhile to investigate the performance of various component analysis methods in the future work. The reconstructed 4D MRI was generated by wrapping the reference image using the remodeled DVFs without considering the MR number difference among the different phases, which may affect the dose calculation. To address this problem, Jacobian transformation matrix can be used to normalize the MR number of the synthetic images.

In this study, we proposed a method to capture regular breathing motion from the noisy DVFs. The remodeled DVFs reconstructed using the linear polynomial fitting model and the PCA could be used to generate ‘synthetic’ 4D MRI with reduced motion artifacts. Moreover, the remodeled DVFs can be further used to generate other 4D images with different purposes by wrapping corresponding reference scans, such as T2w MR, LAVA, and others. It will be very significant for tumor diagnose, planning design, and dose tracking in radiation therapy. It may be of great interest to investigate the possibility of synthesizing T2w 4D MRI with high tumor‐to‐tissue CNR in our future study.

## V. CONCLUSIONS

We have proposed a mathematical method for the reduction of irregular motion artifacts in 4D MR images. The DVFs generated from the DIR was fitted by a linear polynomial fitting model in three temporal and spatial dimensions to correct the potential registration errors introduced by the DIR algorithm. Then the PCA was used to decompose the fitted DVFs into linear combination of principal motion bases, whose spanning subspaces and projections could be used to represent the regular respiratory motion. The ‘synthetic’ MR images at selected phase were generated by deforming the reference MR images using the reconstructed DVFs. Preliminary patient results demonstrated that the proposed method had a potential ability of extracting regular respiratory motion from a patient's 4D MR image set, and restoring distortion of tumor and organs and tissues (such as diaphragm) caused by irregular motion during 4D MR acquisition.

## ACKNOWLEDGMENTS

This work is partly supported by Natural Science Grant of Shandong Province (ZR2010HM010), National Natural Science Foundation of China (81272699), as well as National Natural Science Foundation of China (61201441).

## Supporting information

Supplementary Material
